# miR-10b-5p Suppresses the Proliferation and Invasion of Primary Hepatic Carcinoma Cells by Downregulating EphA2

**DOI:** 10.1155/2021/1382061

**Published:** 2021-12-29

**Authors:** Xu Niu, Haitao Sun, Feng Qiu, Jing Liu, Tianchi Yang, Wei Han

**Affiliations:** ^1^General Surgery, Luhe Hospital, Capital Medical University, Beijing 101100, China; ^2^General Surgery, Tongren Hospital, Capital Medical University, Beijing 101100, China

## Abstract

**Objective:**

To analyze the function of miR-10b-5p in suppressing the invasion and proliferation of primary hepatic carcinoma cells by downregulating erythropoietin-producing hepatocellular receptor A2 (EphA2). *Material and Methods*. Eighty-six hepatic carcinoma (HCC) tissue specimens and 86 corresponding adjacent tissue specimens were collected, and the mRNA expression of miR-10b-5p and Ephrin type-A receptor 2 (EphA2) in the specimens was determined using a reverse transcription-polymerase chain reaction (RT-PCR) assay. Western blot was employed to quantify EphA2, B-cell chronic lymphocytic leukemia/lymphoma-2 (Bcl-2), Bcl-2-associated X protein (Bax), and Caspase-3 in the cells, and CCK8, Transwell assay, and flow cytometry were applied to evaluate the proliferation, invasion, and apoptosis of cells, respectively. Moreover, the dual luciferase reporter assay was utilized for correlation analysis between miR-10b-5p and EphA2.

**Results:**

miR-10b-5p was lowly expressed in HCC, while EphA2 was highly expressed. Cell experiments revealed that miR-10b-5p overexpression or EphA2 knockdown could reduce cell proliferation, accelerate apoptosis, strongly upregulate Bax and Caspase-3, and downregulate Bcl-2. In contrast, miR-10b-5p knockdown or EphA2 overexpression gave rise to reverse biological phenotypes. Furthermore, dual luciferase reporter assay verified that miR-10b-5p was a target of EphA2, and the rescue experiment implied that transfection of pCMV-EphA2 or Si-EphA2 could reverse EphA2 expression and cell biological functions caused by miR-10b-5p overexpression or knockdown.

**Conclusions:**

miR-10b-5p reduced HCC cell proliferation but accelerate apoptosis by regulating EphA2, suggesting it has the potential to be a clinical target for HCC.

## 1. Introduction

Hepatic carcinoma (HCC) is a familiar clinical malignant tumor in the digestive system and is also one of the major reasons for cancer-related death [1]. In recent years, with the changes of social environment and living habits, HCC shows an increasingly higher incidence and mortality [2]. With the progression of medical technology, a considerable progress has been made in the treatment of HCC recently. However, due to the strong invasiveness of HCC cells, the prognosis of most HCC patients after hepatic carcinectomy and intervention embolization is still unsatisfactory [3, 4]. Therefore, it is of great clinical significance to understand the pathogenesis of HCC and uncover new therapeutic targets for HCC patients for the treatment of HCC.

miRNA is a noncoding microRNA, and its role and mechanism in tumors have captured a growing attention over the years [5]. Many studies have been carried out on the role of miRNAs in tumors including HCC. For instance, one study has stated that miR-197-3p can be taken as a prognostic marker and potential treatment target for HCC [6], and one other study has revealed that miR-532-3p can promote the development of HCC by targeting protein tyrosine phosphatase receptor T (PTPRT) [7]. Those studies all imply the strong correlation between miRNA and development and progression of HCC. miR-10b-5p, belonging to the miR-10 family, is located on 2q31.1 chromosome. Some previous studies have reported abnormal expression of miR-10b-5p in tumors such as glioma and renal cell carcinoma [8, 9], and some studies have also found through sequencing abnormal expressed miRNA that miR-10b-5p is a highly dysregulated miRNA in HCC [10]. However, no further research has been conducted on its role and mechanism in the cancer.

We found a targeting relationship between miR-10b-5p and EphA2 through biological information prediction, and Ephrin type-A receptor 2 (EphA2) was reported to be related to the development, metastasis, and prognosis of HCC cells [11]. Therefore, we attempted to investigate the role of miR-10b-5p on the biological functions of HCC cells.

## 2. Materials and Methods

### 2.1. Clinical Data

Eighty-seven patients with primary HCC admitted to our hospital from March 2014 to June 2016 were enrolled, and 87 HCC tissue specimens and 87 corresponding tumor-adjacent tissue specimens were extracted from. The inclusion criteria of the patients were as follows: HCC patients were confirmed according to pathological diagnosis and those with expected survival longer than 3 months. The exclusion criteria of them were as follows: patients with severe infection disease, patients with other comorbid malignant tumors, patients who had received any treated before the experiment, and patients with immune system disorder. All participants and their relatives gave their consent to participate in the experiment and also provided their signed informed consent forms. The experiment was approved by the permission of the Ethics Committee of our hospital.

### 2.2. Experiment Reagents and Materials

Human HCC cell strains (HepG2, BEL-7402, Huh-7, and SMMC-7721) and human normal hepatic cell (HL-7702) from the American Type Culture Collection (ATCC), quantitative reverse transcription-polymerase chain reaction (qRT-PCR), and reverse transcription kit (TransGen Biotech Co., Ltd., Beijing, China), Trizol reagent (Thermo Fisher Scientific-CN), phosphate-buffered saline (PBS) (Gibco Company, United States), dual luciferase reporter gene assay kit (Beijing Biolab Technology Co., Ltd.), CCK-8 kit (Promega Company, the United States), Transwell kit (Costar Company, United States), Annexin V-FITC/PI apoptosis assay kit (Biolab Technology Co., Ltd., Beijing, China), RIPA and BCA kits (Thermo Fisher Scientific, United States), EphA2, Caspase-3, Bax, Bcl-2, and GAPDH antibodies (Cell Signaling Technology), goat anti-rabbit immunoglobulin G (IgG) secondary antibody (BOSTER Biological Technology Co., Ltd., Wuhan, China), electrochemiluminescence (ECL) developer (Thermo Company), and PCR instrument (ABI company, United States). All primers were synthesized by Shanghai Sangon Biotech Co., Ltd., and EphA2 plasmid (pCMV-EphA2) and empty plasmid (pCMV) were synthesized by OriGene (Rockville, Maryland, United States).

### 2.3. qRT-PCR Assay

Total RNA was extracted from collected tissues and cells with a TRIzol kit, and its purity and concentration were determined using an ultraviolet spectrophotometer. Subsequently, 1 *μ*L cDNA was taken from cDNA synthesized by reverse transcription of 5 *μ*g total RNA from tissues and cells, separately, under kit instructions for amplification. Three repeated wells were set for each sample, and the experiment was repeated three times with U6 as an internal reference for miR-10-5p and glyceraldehyde-3-phosphate dehydrogenase (GAPDH) as an internal reference for EphA2. Data in this experiment were analyzed using the 2^-*ΔΔ*CT^. See Table 1 for primer sequences.

### 2.4. Cell Culture and Transfection

HCC cell lines were cultured in Dulbecco's modified Eagle medium (DMEM) with 10% PBS under 5% CO_2_ at 37°C. Upon reaching 85% confluency in adherent growing, the cells were digested with 25% trypsin and then cultured in the medium for passage. miR-10b-5p-mimics (overexpression sequence), miR-10b-5p-inhibitor (inhibition sequence), miR negative control (miR-NC), targetedly inhibited EphA2 (si-EphA2), negative control RNA (Si-NC), EphA2 plasmid (pCMV-EphA2), and empty plasmid (pCMV) were transfected into cells using a Lipofectamine 2000 kit, separately, in strict accordance with the kit instructions.

### 2.5. Western Blot Assay

The RIPA lysis method was applied to lyse cells to extract the total protein, and the concentration of the extracted protein was determined using the BCA method. With concentration adjusted to 4 *μ*g/*μ*L, the protein was subject to sodium dodecyl sulfate-polyacrylamide gel electrophoresis (SDS-PAGE) and then transferred to a PVDF membrane. Afterwards, the membrane was cultured with EphA2 (1 : 500), Caspase-3 (1 : 500), Bax (1 : 500), Bcl-2 (1 : 500), and GAPDH (1 : 1000) at 4°C for one night after being sealed with 5% skim milk for 2 h. The membrane was washed to remove the primary antibody, added with horseradish peroxidase-labeled goat anti-rabbit secondary antibody (1 : 1000), cultured at 37°C for 1 h, and rinsed with PBS three times, 5 min each time. Then, the membrane was made to be luminescent with ECL and developed.

### 2.6. Cell Proliferation Assay

The proliferation ability of HepG2 and Huh-7 cells was evaluated by a CCK-8 kit. After being transfected for 48 hours, the cells were collected and diluted to 3 × 10^4^ cell/mL and transferred to a 96-well plate at 100 *μ*L per well. The plate was cultured under 5% CO_2_ at 37°C, and then, 10 *μ*L CCK8 solution was added into each well at 0 h, 24 h, 48 h, and 72 h after adherent growth of the cells. After addition of the solution, the plate was continuously cultured at 37°C for 2 h each time, and the optical density of each well at 450 nm was analyzed using an enzyme mark instrument to analyze proliferation of the cells and draw growth curves of the cells. The experiment was tripled.

### 2.7. Transwell Assay

After being transfected for 24 hours, the cells were transferred to a 24-well plate at 3∗10^3^ cells/well, digested with trypsin, and then transferred to the upper compartment, followed by addition of 200 *μ*L RPMI 1640. RPMI1640 with 10% FBS was put into the lower compartment. Afterwards, the chamber was cultured at 37°C for 48 h, and the substrates and cells not penetrating the microporous membrane were wiped off. The membrane was washed with PBS three times, immobilized with paraformaldehyde for 10 min, and washed with double distilled water three times again, and it was then stained with 0.5% crystal violet after being dried out. Finally, cell migration was analyzed using a microscope.

### 2.8. Apoptosis Assay

The transfected cells were trypsinized with 0.25% trypsin. After it, the cells were washed with PBS twice and then added with 100 *μ*L binding buffer to prepare 1∗10^6^ cells/mL suspension. Annexin V-FITC and PI were put into the suspension in order, and the suspension was cultured in the dark at indoor temperature for 5 min and then detected using the FACS Verse flow cytometer system. The experiment was tripled, and the data were averaged as results.

### 2.9. Dual Luciferase Assay

The EphA2-3′UTR wild-type (Wt) and EphA2-3′UTR mutant type (Mut) as well as miR-10b-5p-mimics, miR-10b-5p-inhibitor, and miR-NC were transferred into HepG2 and Huh-7 cells by a Lipofectamine 2000 kit. After transfection for 48 hours, the luciferase activity of the cells was measured with a dual luciferase reporter gene assay kit (Promega).

### 2.10. Statistical Analysis

In this study, the collected data were analyzed statistically using SPSS20.0 and visualized into required figures using GraphPad 7. Comparison between groups was conducted using the independent *t*-test, and multigroup comparison was carried out using the one-way ANOVA. Post hoc pairwise comparison was carried out using the LSD *t*-test. Pearson's correlation was conducted for correlation analysis between miR-10b-5p and EphA2. *p* < 0.05 implies a significant difference.

## 3. Results

### 3.1. Reduction of miR-10b-5p in HCC Tissues and Cells

The RT-PCR assay revealed that compared with tumor-adjacent tissues and normal hepatic cells, HCC tissues and cells showed a great decrease in the expression of miR-10b-5p (*p* < 0.05) and an increase in the expression of EphA2 (*p* < 0.05), and the expression of miR-10b-5p was negatively related to that of EphA2 (*r* = −0.698, *p* < 0.05). ROC curves indicated that the area-under-the-curve of miR-10b-5p in diagnosing HCC was 0.937 (*p* < 0.05) (Figure 1).

### 3.2. Influences of miR-10b-5p on Biological Functions of HCC Cells

Compared with HepG2 and Huh-7 cells transfected with miR-10b-5p-mimics, those transfected with miR-NC showed a great increase in the expression of miR-10b-5p, while those transfected with miR-10b-5p-inhibitor showed a great decrease in it. The detection of the biological functions of cells in the two groups revealed that compared with the miR-NC group, the cells transfected with miR-10b-5p-mimics showed significantly weakened proliferation and invasion abilities and significantly increased apoptosis rate, while those transfected with miR-10b-5p-inhibitor showed significantly strengthened proliferation ability and significantly decreased apoptosis rate. In addition, compared with the miR-NC group, cells transfected with miR-10b-5p-mimics showed significantly downregulated Bcl-2 and significantly upregulated Caspase-3 and Bax, while those transfected with miR-10b-5p-inhibitor showed significantly upregulated Bcl-2 and significantly down-regulated Caspase-3 and Bax (Figure 2).

### 3.3. Influences of EphA2 on the Biological Functions of HCC Cells

Compared with HepG2 and Huh-7 cells transfected with Si-EphA2, those transfected with Si-NC presented a great decrease in the expression of EphA2, while those transfected with pCMV-EphA2 showed a great increase in the expression of EphA2. Detection of the biological functions of cells in the two groups revealed that compared with the Si-NC group, cells transfected with Si-EphA2 showed significantly weakened proliferation and invasion abilities and significantly increased apoptosis rate, significantly downregulated Bcl-2, and significantly upregulated Caspase-3and Bax. In addition, compared with the pCMV group, cells transfected with pCMV-EphA2 showed significantly strengthened proliferation and invasion abilities, significantly weakened apoptosis, significantly upregulated Bcl-2, and significantly downregulated Caspase-3 and Bax (Figure 3).

### 3.4. Dual Luciferase Reporter Assay

In order to further understand the correlation of miR-10b-5p with EphA2, Targetscan 7.2 was utilized to predict downstream target genes of miR-10b-5p, and it was found that there was a targeted binding locus between EphA2 and miR-10b-5p. To confirm it, we carried out a dual luciferase reporter assay, finding that overexpression of miR-10b-5p strongly lowered the luciferase activity of EphA2-3′UTR Wt (*p* < 0.05) but exerted no effect on that of EphA2-3′UTR Mut (*p* > 0.05). The western blot (WB) assay revealed that transfection of miR-10b-5p-mimics greatly decreased the expression of Rap1b in HepG2 and Huh-7 cells and transfection of miR-10b-5p-inhibitor greatly lowered it in the cells (both *p* < 0.05) (Figure 4).

### 3.5. Rescue Experiment

miR-10b-5p-mimics+pCMV-EphA2 or miR-10b-5p-inhibitor+Si-EphA2 was cotransfected into HepG2 and Huh-7 cells, and it came out that cotransfection with pCMV-EphA2 reversed the downregulation of EphA2 caused by overexpression of miR-10b-5p and cotransfection of Si-EphA2 also reversed the upregulation of it caused by ablating miR-10b-5p. Moreover, detection of biological functions revealed that EphA2 could reverse the influence of miR-10b-5p on the proliferation, invasion, and apoptosis of HCC cells (Figure 5).

## 4. Discussion

HCC is a malignant tumor with high incidence. Its symptoms are usually insidious, so most patients have already missed the optimal treatment opportunity at the time of diagnosis, causing unfavorable prognosis [11]. Many studies have reported the dysregulation of miRNA in HCC, and they believe that dysregulation of miRNA and its functions as an oncogene or tumor suppressor gene are one of the main driving forces for HCC [12, 13]. Therefore, it is of great significance to identify the function and functional mechanism of miRNA in HCC for diagnosis and treatment of the cancer.

miR-10b-5p has been proved to play different roles in different tumors. For instance, the expression of it decreased in breast cancer and increased in colorectal cancer [14, 15]. However, the expression of miR-10b-5p in HCC and relevant mechanisms are still under investigation. In our study, it was found that the expression of miR-10b-5p in HCC tissues and cells decreased, and ROC curves revealed the high diagnostic value of miR-10b-5p in the disease. One study has stated that miR-10b-5p is able to inhibit the proliferation of glioma and terminate the cell cycle [16]. In our study, we uncovered that overexpression of miR-10b-5p could strongly hinder the invasion and proliferation of HCC cells and accelerate apoptosis of them, while reducing miR-10b-5p would give rise to opposite results, which suggested that miR-10b-5p acted as a tumor suppressor gene in HCC. One previous study has also found reduced miR-10b-5p in colorectal cancer patients under liver metastasis [17]. However, there are no more demonstrations on the functional mechanism of miR-10b-5p in HCC, so for the purpose of further exploring the mechanism, we have predicted targeting relationship between EphA2 and miR-10b-5p based on the biological information website Targetscan.

EphA2 is one of the members of receptor tyrosine kinase, and it has been reported to be crucial in the proliferation, metastasis, and growth of tumors [18]. EphA2 showed overexpression in HCC tissues and cells in our study, and it was regulated in various cancers including gastric cancer and lung cancer according to some studies [19, 20]. In order to further verify the influences of EphA2 on HCC cells, we regulated EphA2 expression in HCC cells, and it came out that downregulation of EphA2 expression strongly inhibited the invasion and proliferation of HCC cells. We also transfected plasmids of EphA2 into HCC cells, finding that after transfection, the invasion and proliferation of HCC cells were strengthened and the apoptosis of it was weakened. These results suggested that EphA2 played a role of oncogene in HCC. One previous study has concluded that downregulation of EphA2 in HCC cells can inhibit cell invasion [21], which is consistent with our results. Moreover, one study has reported the relation between EphA2 and the metastasis and prognosis of HCC [22], and one other study has pointed out that miR-26a can suppress the migration and invasion of HCC cells by downregulating EphA2 [23]. These studies further illustrate the role of EphA2 in HCC. In our study, correlation analysis revealed the negative correlation between miR-10b-5p and EphA2, and the dual luciferase reporter assay further verified the targeting correlation between them. In order to further verify that miR-10b-5p affects HCC cells by regulating EphA2, we carried out a rescue experiment, finding that pCMV-EphA2 could reverse the downregulation of EphA2 and influences on biological functions caused by overexpression of miR-10b-5p, and Si-EphA2 could reverse the upregulation of EphA2 and influences on cells caused by inhibition of miR-10b-5p, which further proved that miR-10b-5p exerted its effect on HCC cells by regulating EphA2. As far as I know, this is the first time that we have proved that miR-10b-5p can inhibit the expression of EphA2 to affect the invasion, proliferation, and apoptosis of HCC cells.

## 5. Conclusion

miR-10b-5p can suppress the invasion and proliferation of primary HCC cells and accelerate apoptosis of them by downregulating EphA2, so it has the potential to be a target for diagnosis and treatment of HCC. However, there are still some deficiencies in this study. For example, we have not conducted any animal experiments to further verify the role of miR-10b-5p in vivo. Secondly, we have not conducted any experiments on the downstream mechanism of EphA2. In the future, we will further improve our experiments to provide support for our conclusions with more data.

## Figures and Tables

**Figure 1:** Expression of miR-10b-5p in HCC tissues and cells. (a) Expression of miR-10b-5p in HCC tissues. (b) Expression of EphA2 mRNA in HCC cells. (c) Expression of miR-10b-5p in HCC cells. (d) Expression of EphA2 mRNA in HCC cells. (e) ROC curves of miR-10b-5p for HCC. (f) Correlation between miR-10b-5p and EphA2. ∗ indicates *p* < 0.05.

**Figure 2:** Influences of miR-10b-5p on the biological functions of HCC cells. (a) Expression of miR-10b-5p in transfected cells. (b) Influences of miR-10b-5p on the proliferation ability of HCC cells. (c) Influences of miR-10b-5p on the invasion ability of HCC cells. (d) Influences of miR-10b-5p on the apoptosis rate of HCC cells. (e) Influences of miR-10b-5p on apoptosis-related proteins in HCC cells. ∗ indicates *p* < 0.05.

**Figure 3:** Influences of EphA2 on the biological functions of HCC cells. (a) Expression of EphA2 mRNA in transfected cells. (b) Influences of EphA2 on the proliferation ability of HCC cells. (c) Influences of EphA2 on the invasive ability of HCC cells. (d) Influences of EphA2 on the apoptosis of HCC cells. (e) Influences of EphA2 on apoptosis-related proteins in HCC cells. ∗ indicates *p* < 0.05.

**Figure 4:** Dual luciferase reporter assay. (a) Influences of miR-10b-5p on dual luciferase activity of EphA2. (b) Influences of miR-10b-5p on EphA2. ∗ indicates *p* < 0.05.

**Figure 5:** Rescue experiment. (a) Expression of EphA2 mRNA in co-transfected cells. (b) Influences of cotransfection on the proliferation ability of HCC cells. (c) Influences of cotransfection on the invasion ability of HCC cells. (d) Influences of cotransfection on the apoptosis of HCC cells. (e) Influences of cotransfection on apoptosis-related proteins of HCC cells. ∗∗ indicates that in comparison of other groups, *p* < 0.05; ∗ indicates *p* < 0.05.

**Table 1:** Primer sequences.

Factor	Upstream sequence	Downstream sequence
miR-10b-5p	5′-GGGTACCCTGTAGAACCG-3′	5′-AACTGGTGTCGTGGAGTCGGC-3′
U6	5′-CTCGCTTCGGCAGCACA-3′	5′-AACGCTTCACGAATTTGCGT-3′
EphA2	5′-GGGACCTGATGCAGAACATC-3′	5′-AGGCATTTCACTCACAGGGG-3′
GAPDH	5′-GGAGTCAACGGATTTGGT-3′	5′-GTGATGGGATTTCCATTGAT-3′

## Data Availability

The data used during the present study are available from the corresponding author upon reasonable request.

## References

[1] Nakagawa H., Fujita M., Fujimoto A. (2019). Genome sequencing analysis of liver cancer for precision medicine. *Seminars in Cancer Biology*.

[2] Melkonian S. C., Jim M. A., Reilley B. (2018). Incidence of primary liver cancer in American Indians and Alaska Natives, US, 1999-2009. *Cancer Causes & Control*.

[3] Colombo J., Jardim-Perassi B. V., Ferreira J. P. S. (2018). Melatonin differentially modulates NF-*к*B expression in breast and liver cancer cells. *Anti-Cancer Agents in Medicinal Chemistry*.

[4] Cast A., Valanejad L., Wright M. (2018). C/EBP*α*-dependent preneoplastic tumor foci are the origin of hepatocellular carcinoma and aggressive pediatric liver cancer. *Hepatology*.

[5] Callegari E., Domenicali M., Shankaraiah R. C. (2019). MicroRNA-based prophylaxis in a mouse model of cirrhosis and liver cancer. *Molecular Therapy-Nucleic Acids*.

[6] Ni J. S., Zheng H., Huang Z. P. (2019). MicroRNA-197-3p acts as a prognostic marker and inhibits cell invasion in hepatocellular carcinoma. *Oncology Letters*.

[7] Wang Y., Yang Z., Wang L. (2019). miR-532-3p promotes hepatocellular carcinoma progression by targeting _PTPRT_. *Biomedicine & Pharmacotherapy*.

[8] Li W., Li C., Xiong Q., Tian X., Ru Q. (2019). MicroRNA-10b-5p downregulation inhibits the invasion of glioma cells via modulating homeobox B3 expression. *Experimental and Therapeutic Medicine*.

[9] Li Y., Chen D., Li Y. (2016). Oncogenic cAMP responsive element binding protein 1 is overexpressed upon loss of tumor suppressive miR-10b-5p and miR-363-3p in renal cancer. *Oncology Reports*.

[10] Wojcicka A., Swierniak M., Kornasiewicz O. (2014). Next generation sequencing reveals microRNA isoforms in liver cirrhosis and hepatocellular carcinoma. *The International Journal of Biochemistry & Cell Biology*.

[11] Hiraoka A., Kumada T., Michitaka K., Kudo M. (2019). Newly proposed ALBI grade and ALBI-T score as tools for assessment of hepatic function and prognosis in hepatocellular carcinoma patients. *Liver Cancer*.

[12] Dong H., Wang J., Yang Y. (2018). Overexpression of miR-451a inhibits cell proliferation by targeted macrophage migration inhibitory factor in HepG2 cells. *Xi Bao Yu Fen Zi Mian Yi Xue Za Zhi*.

[13] Liu B., Yang X. F., Liang X. P. (2018). Expressions of MiR-132 in patients with chronic hepatitis B, posthepatitic cirrhosis and hepatitis B virus-related hepatocellular carcinoma. *European Review for Medical and Pharmacological Sciences*.

[14] Wang J., Yan Y., Zhang Z., Li Y. (2019). Role of miR-10b-5p in the prognosis of breast cancer. *PeerJ*.

[15] Schee K., Lorenz S., Worren M. M. (2013). Deep sequencing the microRNA transcriptome in colorectal cancer. *PLoS One*.

[16] Gabriely G., Yi M., Narayan R. S. (2011). Human glioma growth is controlled by microRNA-10b. *Cancer Research*.

[17] Liu J., Li H., Sun L. (2019). Epigenetic alternations of microRNAs and DNA methylation contribute to liver metastasis of colorectal cancer. *Digestive Diseases and Sciences*.

[18] Sulman E. P., Tang X. X., Allen C. (1997). _ECK,_ a human _EPH_ -related gene, maps to 1p36.1, a common region of alteration in human cancers. *Genomics*.

[19] Tang L., Hu H., He Y. (2018). The relationship between miR-302b and EphA2 and their clinical significance in gastric cancer. *Journal of Cancer*.

[20] Ishigaki H., Minami T., Morimura O. (2019). EphA2 inhibition suppresses proliferation of small-cell lung cancer cells through inducing cell cycle arrest. *Biochemical and Biophysical Research Communications*.

[21] Jin R., Lin H., Li G. (2018). TR_4_ nuclear receptor suppresses HCC cell invasion via downregulating the EphA2 expression. *Cell Death & Disease*.

[22] Yang P., Yuan W., He J. (2009). Overexpression of EphA2, MMP-9, and MVD-CD34 in hepatocellular carcinoma: implications for tumor progression and prognosis. *Hepatology Research*.

[23] Li H., Sun Q., Han B., Yu X., Hu B., Hu S. (2015). MiR-26b inhibits hepatocellular carcinoma cell proliferation, migration, and invasion by targeting EphA2. *International Journal of Clinical and Experimental Pathology*.

